# Understanding Physical Activity and Exercise Behavior in China University Students: An Application of Theories of the Flow and Planned Behavior

**DOI:** 10.1155/2022/7469508

**Published:** 2022-05-19

**Authors:** Haitao Feng, Jin Hwang, Li Hou

**Affiliations:** ^1^Hebei University of Science and Techology, Shijiazhuang 050018, China; ^2^Jeonbuk National University, Jeonju 54896, Republic of Korea; ^3^Shandong Sport University, Jinan 250102, China

## Abstract

**Objectives:**

The purpose of this study was to examine a extended model of the theory of planned behavior (TPB) model by adding the variables of the flow theory and to investigate Chinese university students' exercise behavior and its influence factors.

**Methods:**

The hypothesized model was validated through testing three competing models using a sample collected from 248 Chinese university students involving 165 males and 83 females.

**Results:**

The three competitive models fitted well and predicted exercise behavior significantly. Among them, the enjoyment + TPB model is the optimal model.

**Conclusions:**

Enjoyment and concentration can all predicting exercise behavior directly or indirectly. Enjoyment is stronger than concentration in predicting TPB constructs and exercise behavior, and it is a more important predictor than concentration in the field of exercise behavior research. *Values*. Research provides insights to better understand the exercise behavior of Chinese university students as well as useful information for designing exercise interventions and developing university students' education and training.

## 1. Introduction

### 1.1. Necessary of the Research

According to the report of Sohu news in 2017, during the military training of Peking University students, nearly 3,500 students received more than 6,000 medical visits, and especially in the first week, many people fainted. To some extent, this reflects the serious problems of university students' physique. In addition, according to the test results of the national students' physique health survey, in 2010 and 2015, compared with 2005, the overall decline in the physical fitness of Chinese university students has not been alleviated. The 2020 Chinese university Student Health Survey also reports a lots of health problems such as the skin condition, poor sleep quality, poor mood, obesity, and other health problems. What is more serious is the events of sudden death of university students during sports activities.

In the above situation, a lack of physical exercise is undoubtedly the main reason. The survey of university students shows that nearly 70% of university students fail to meet the adult physical exercise health standards, and some of them only take part in physical exercise during the sports standards test. Because the willing of the current university students to participate in physical activity is not high and the motivation is generally not strong, it is particularly urgent to draw lessons from exercise psychology of scientific and to explain, predict, and intervene the physical activity and exercise behavior of the university students [1, 2].

#### 1.1.1. Flow

Flow is one of the psychological theories, evidenced to be related to intrinsic motivational factors [3]. It is defined as “the holistic sensation that people feel when they act with total involvement and the experience is so enjoyable that people will do it even at great cost, for the sake of doing it” [4]. Studies have shown that flow may have an important role to play in the adoption and maintenance of health-promoting behaviors in university students [5], also may improve the quality of their experiences, and promote exercise adherence(dimensions relating to concentration and self-transcendence) [6], as well as to foster their exercise behavior(dimensions relating to clear goals, concentration, and autotelic experience) [7]. Flow has increasing potential in exercise and physical activity promotion given the importance of positive experiences for long-term participation [8]. As such, flow is highly relevant in sport and exercise [9].

#### 1.1.2. The Theory of Planned Behavior

The theory of planned behavior is a psychological theory that links beliefs to behavior. The theory maintains that three core components, namely, attitude, subjective norms, and perceived behavioral control, together shape behavioral intentions of an individual. In turn, behavioral intention is the most proximal determinant of human social behavior (from Wikipedia). The theory of planned behavior [10] is a leading framework to examine exercise behavior [1,11]. It has been applied to the prediction of a wide range of social and health behaviors (for reviews, see [2,12]), including exercise [11,13]. In their meta-analysis of 72 theory of planned behavior-exercise studies, Hagger and his colleagues [11] reported significant average correlations between the attitude (*r* = .48), subjective norm (*r* = .25), and perceived behavioral control (*r* = .44) constructs and exercise intentions. Together, these variables explained 45% of the variance in exercise intentions. Both intention (*r* = .42) and perceived behavioral control (*r* = .31) were found to have significant average correlations with exercise behavior, explaining 27% of the variance in exercise behavior.

Since then, scholars in the field of physical exercise behavior have continued to explore how to improve the prediction effect of the theory of planned behavior and how to explore the interaction mechanism between theory of planned behavior and other sociological and psychological factors. Some studies have extended the theory of planned behavior theoretical framework by adding new variables including self-efficacy and past behavior (Lijuan Wang and Ying ZhanG) [14], relative intention (Gao Guangjian, Wu Zhouyang, and Guo Lu [15]), action control and emotion (Zhang Wenjuan and Mao Zhixiong [16]), online social support [17], exercise intensity preference and exercise intensity tolerance [18], SDT [19,20], perceived risks, and past experience [21], and habit [22] to improve the predictive effect of the theory of planned behavior on exercise behavior. The research has achieved some results, but there are still some regrets.

#### 1.1.3. The Feasibility of the Integration of the Two Theories

The theory of planned behavior assumes that an individual's behavior is reasoned, controlled, and planned, whether or not an intention translates into an action depends on an individual's motivation and how much energy they are willing to invest. Although previous researchers have found the theory of planned behavior to be a sound model for understanding the intention-behavior relationship [23–27], it is clear that the theory of planned behavior is better able to explain exercise intentions than behavior. Such inconsistencies imply that there may be other factors that influence exercising behaviors. Ajzen [10] concedes, “the Theory of Planned Behavior is, in principle, open to the inclusion of additional predictors if it can be shown that they capture a significant proportion of the variance in intentions or behavior after the theory's current variables have been taken into account.” This suggests the model is open to the inclusion of further variables that may capture additional variance in behavior. Variables external to the theory of planned behavior framework may have effects on behavior and intention through the constructs of attitude, subjective norm, and perceived behavioral control [28,29]. That is, variables external to the theory of planned behavior are potential antecedents to the formation of social cognitions.

Flow factors have been added into the theory of planned behavior framework to capture emotional factors (intrinsic motivation) and improved the prediction effect of behavior and intention that have shown the efficacy [30,31]. Chen and Chen [31] have applied flow factors enjoyment and concentration to predict individual riding intention and behaviors by the part media effect of attitude. Charles Atombo, Chaozhong Wu, Hui Zhang, and *Tina* D. Wemegah [30] added enjoyment and concentration into the TBP model to predict speeding intention and behavior by the partial media effect of attitude, subjective norm, and perceived behavioral control. Ahmed Ibrahim Alzahrani, Imran Mahmud, T. Ramayah, Osama Alfarraj, and Nasser Alalwan [19] extended the theory of planned behavior by enjoyment to explain online game playing behavior through the partial media effect of attitude. Sang M. Lee and Liqiang Chen [32]'s study shows that flow influences online consumer behavior through several important latent constructs (concentration, enjoyment, time distortion, telepresence) by the partial media effect of attitude and perceived behavioral control. Research examined flow and its effects on online consumer behavior in a unified model, which draws upon the theory of planned behavior.

So, it can be seen from the view above, and in general, within the theory of planned behavior framework, flow mainly affects intention and behavior through several important factors（Sang M. Lee and Liqiang Chen [32], and enjoyment and concentration are used most and have relatively high reliability. Enjoyment is described by Csikszentmihalyi as an activity whose final objective is the experience itself, which is carried out not for the hope of some future benefit, but simply because the activity in itself is the reward. It constitutes one of the most representative factors of flow—optimal and momentary experience in which the person is absorbed in a specific activity, feeling great enjoyment—favoured by intrinsic motivation for which the level of individual skill and the difficulty of the task are combined. Concentration has been described as receptive attention that may be reflected in a sustained consciousness of ongoing events and experiences that narrow the focus of awareness [4]. Concentration only allows a very select range of information into awareness [4]. Charles Atombo, Chaozhong Wu, Hui Zhang, and *Tina* D. Wemegah [30] believed that the flow theory provides enjoyment and concentration as two major factors impacting on individual intentions and behaviors [31,33]. Enjoyment and concentration may directly influence intention and behavior, and may also indirectly influence intention and behavior through the partial mediation of the theory of planned behavior factors-attitude, subjective norm, and perceived control. In international sport and exercise research field, flow is commonly understood in terms of nine dimensions (e.g., [34]). The ninth dimension autotelic experience (i.e., flow is described as rewarding and enjoyable) implied the enjoyment and in China, and the autotelic experience as the ninth dimension of flow is translated directly as 享受, which is exactly the same with enjoyment [35]. Jackson and Csikszentmihalyi [34] said that autotelic experience is the flow dimension most closely aligned to intrinsic motivation.

So far, in conclusion, some progress has been made in the study of interpretation of exercise behavior-based the theory of planned behavior, but the “gap” between the interpretation effect of intention and behavior has not been completely solved. For now, it seems to be a good idea to integrate flow with the theory of planned behavior. But the nature of the roles and interplay, of flow constructs within the theory of planned behavior framework when attempting to explain the determinants of motivations for intention to exercise and exercise behavior, is not yet seen and known. On the basis of Ajzen recommendations, because TPB and flow are two completely different theories, the combination of the two theories should enable us to deepen our understanding of the relationship between intention and behavior of motion.

#### 1.1.4. Purpose of the Research

Thus, this study aims at putting the enjoyment and concentration—two factors of flow into the theory of planned behavior framework and to construct competing models in explaining Chinese university students' intention to exercise and exercise behavior so as to verify whether the integrated model can improve the predictive power of exercise intention and behavior, and to investigate the interaction mechanism between flow factors and theory of planned behavior factors in the integrated model and to evaluate which factors are important for explaining intention and behavior of exercise. The result of this study can provide theoretical reference for promoting the exercise behavior of Chinese university students and enrich the psychological theory of physical exercise research.

#### 1.1.5. Exercise Behavior and Physical Activity

Exercise behavior is a planned, structured, and repetitive form of physical activity, which is performed to improve or maintain physical fitness [36]. Physical activity was defined as “any bodily movement produced by skeletal muscles that requires energy expenditure” [36]. This definition encompasses any daily life activity from occupational, household, and other daily tasks to sports and exercise behavior. Because the low-intensity physical activity and exercise behavior has little significance to the physical health of university students [37], physical activity and exercise behavior were defined in this study for all participants as activities performed at a moderate to vigorous intensity for at least 30 min each time per week [14]. Participants were asked to use this definition when answering all exercise-related questions.

### 1.2. Hypothesis of Research

Due to the previous studies on exercise intention and behavior based on the theory of planned behavior (Hagger et al. [11]), we posit the following:

 
**H1:** Theory of planned behavior factors (attitude, subjective norm, and perceived behavioral control) positively and directly predict exercise intention and predict exercise behavior indirectly through exercise intention.
  Gardner and his colleagues [38] support the use of enjoyment and behavioral intentions as indicators of sport participation/dropout behavior. Kathleen A. Ginis et al. [39] found enjoyment-mediated changes in attitudes toward physical activity. His finding bolsters notion that affective reactions to an object or an action can shape attitudes toward it [40]. The observed mediational relationship between exercise, enjoyment, and attitudes suggests that there is utility in the further study of enjoyment within a theory of planned behavior framework. So, we posit the following:
 
**H2:** Enjoyment positively predicts exercise attitude, exercise intention, and behavior.
  Dishman and his colleagues [41] believed that an indirect effect of exercise enjoyment on exercise through an influence on self-efficacy. This explanation is consistent with Dishman and his colleagues' [42] finding that enjoyment's effects on physical activity are mediated partially by changes in self-efficacy, a control construct that is conceptually similar to PBC [43]. Therefore, in an enjoyment disposition, if an exerciser has a strong intention to perform an exercise behavior, he may feel to have the necessary resources and skills to perform the behavior [44]. In other words, enjoyment increases a person behavioral control and has a positive predictive effect on perceived behavior control [32]. So, we posit the following:
 
**H3:** Enjoyment positively predicts perceived behavior control.
  Research studies examining relationship between enjoyment, intention, and behavior through subjective norm are seldom. Nevertheless, Charles Atombo and his colleagues [30] believe that drivers' tendency to speed in the enjoyment state is influenced by the subjective norms of important individuals (e.g., family, friends, spouse, police) that is subjective norms [45]. Similarly, in physical exercise, the enjoyment of this positive emotional experience can be influenced by the opinions of the important people around you. On the basis of these, we hypothesize that the following:
 
**H4:** Enjoyment positively predicts subjective norm.
  Similarly with enjoyment, the concentration has been established to be positively related to attitude and intention [31]. It may be based on the facts that individuals are more likely to be motivated to continue or repeat any activity that is enjoyable as compared to the same activity that is not enjoyable. Moreover, in the pursuit of a goal, a person must concentrate on the task and forget everything [46]. All these studies have evidenced that flow constructs are capable of predicting intention and behavior. A current study also examined the causal relationship between flow constructs and PBC [32] and found concentration to be positively related to PBC constructs (self-efficacy and controllability). A person's concentration could also affect exercise intentions and behavior when perceived other important people are against or in support of exercise [44]. Therefore, we hypothesize that the following
  H5: Concentration is positively related to attitude, subjective norm, PBC, intention, and exercise violation behavior.

To sum up, we build the integration model as shown in Figure 1.

## 2. Research Methods

### 2.1. Participants

The object of this study is 248 Chinese university students from 5 Universities of Hebei province, China: Hebei University, Hebei University of Science and Technology, Hebei University of Economics and Business, Shijiaz tiedao University, and Shijiazhuang University. In order to collect data, the purpose and contents of the research were explained to the student administrator of 5 universities and the prior consent of the questionnaire was obtained. Of the 255 questionnaires recovered, those that were deemed untrue were reviewed, and 248 questionnaires were used in the final analysis after the exclusion of 7 questionnaires. There were 165 males (66.5%) and 83 females (33.5%), 112 coming from city and 136 coming from country, 55 in grade 1 (22.2%), 92 in grade 2 (37.1%), 64 in grade 3(25.8%), and 37 in grade 4(14.9%). All the research objects are ordinary university students with nonsports major and nonsports background, as shown in Table 1.

### 2.2. Measures

#### 2.2.1. Flow Scale

The flow questionnaire (FSS) was rewritten by Marsh and Jackson [47] based on Csikszentmihalyi [48]'s immersion experience factors to measure the state of immersion experienced by sports participants in physical activity situations. The questionnaire used in this study was composed of two subfactors including enjoyment and concentration. The main questionnaire consists of 4 questions for enjoyment and 4 questions for concentration. The criteria for all questions ranged from “Never experienced (1)” to “Always experienced (7).” The Cronbach's *α* coefficient is 0.89, indicating a high degree of scale reliability.

#### 2.2.2. Theory of Planned Behavior Scale

Theory of planned behavior scales have been used previously in physical activity research with similarly aged adolescents, and they have established an acceptable reliability [14, 49]. In this study, intention to perform exercise behavior was assessed by the following three items: (1) “I plan to do physical activities that make me out of breath for at least three or more times during my free time in the next week”; (2) “I expect to do physical activities that make me out of breath during my free time in the next week”; and (3) “I intend to do physical activities that make me out of breath for at least three or more times during my free time in the next week.” Responses were given using a scale ranging from 1 (unlikely) to 7 (likely). Attitude towards performing exercise behavior in the subsequent week was assessed by the item: “My doing physical activities at least three or more times in the next week is. . .,” using three scales, namely, good-bad, exciting-boring, and fun-unpleasant. Subjective norm was measured by a seven-point scale that ranged from 1(strongly disagree) to 7 (strongly agree). A single item was included in this section, “Most people important to me think I should do physical activities that make me out of breath at least three or more times in the next week.” The phrase “out of breath” instead of “moderate to vigorous” was used to ensure that the participants understand the type of physical activity under investigation. The phrase has been successfully used in previous research with adolescents [11,49]. The Cronbach's *α* coefficient is 0.89, indicating a high degree of scale reliability.

#### 2.2.3. Physical Activity and Exercise Behavior Scale

Physical activity and exercise behavior were measured by the Godin Leisure Time Exercise Questionnaire (GLTEQ) [50]. The GLTEQ has been shown to produce test-retest reliable and valid scores with children and adolescents [51]. In this study, participants were asked to recall the number of times in the previous week that they usually participated in at least 30 min of mild, moderate (not exhausting), and strenuous (characterized by rapid heartbeats) physical activity during their free time. Examples of different intensities of physical activity were provided to help participants gain a better understanding of the concepts of physical activity. The participants' answers for strenuous and moderate exercise were then multiplied by 9 and 5 METs (metabolic equivalent of energy), respectively [50], and the scores were added to obtain the overall METs score.

### 2.3. Data Analysis

After the questionnaire was collected, the initial screening of the questionnaire was carried out. Delete the questionnaires that clearly do not meet the requirements. Then, the rest of the questionnaire data were sorted and coded, and the normal distribution test was carried out. And then, the data were been coded and analyzed by SPSS 25.0.

Analyze data according to the structural equation model analysis method proposed by Anderson and Gerbing [52]. The first step is to conduct confirmatory factor analysis to verify the psychometric attributes of the measurement model to ensure that the measured variables reliably reflect the latent variables. In the second step, structural equation model estimation is performed on the theoretical model to determine the adequacy of the model construction and test the hypothesis. Using various fit indices to check the structural models, as follows: adjusted goodness-of-fit index (AGFI), goodness-of-fit index (GFI), root mean square error of approximation (RMSEA), and comparative fit index (CFI). According to Hair and his colleagues' opinion (2006), values of AGFI, GFI, and CFI of 0.9 or above and RMSEA of 0.08 or less all show a good fit between the data and the model. The statistical software of AMOS24 will be used to analyze the data in this study.

### 2.4. Reliability and Validity Test

In order to further determine whether the selected questionnaire is suitable for the research needs, questionnaires will be tested for structural reliability and validity.

1. Common method bias test. The scales used were all from abroad, and the survey objects were Chinese university students, so a common method bias test was required. First, backtranslation is used to test the equivalence of the language. We asked Chinese and English language experts for translation and back translation, respectively, carefully compared the translation with the original text, and made repeated reviews based on the opinions of relevant experts. Then, we sent the draft to three English and Chinese experts in the field of physical education to identify the validity of the content and found no significant changes in meaning. There were no major changes. Fifteen ordinary college students were invited to fill in the Chinese questionnaire. The feedback scale of students was clear and easy to understand. During data analysis, in addition to confirmatory factor analysis and reliability test for each scale, Harman single-factor method recommended by Podsakoff was used to check common method bias. Unrotated principal component factor analysis showed that all items had 5 common factors with characteristic root values greater than 1, and the first factor explained 21.55% of variance. Less than 40% indicates that the questionnaire common method bias of the study is not serious.
2. Confirmatory factor analysis had been implemented and carried out to check the fit of the factor models to ensure that the measurement variables reliably reflect the latent variable before proceeding to test the structural model. The goodness-of-fit indices of flow include *χ*2 = 35.267, df = 247, *χ*2/df = 1.856, GFI = 0.957, and IFI = 0.980, NFI = 0.957, CFI = 0.979, RMSEA = 0.059, and the goodness-of-fit indices of TPB include *χ*2 = 53.960, df = 247, *χ*2/df = 1.927, GFI = 0.976, and IFI = 0.988, NFI = 0.976, CFI = 0.988, RMSEA = 0.061. Most of these indices are all within the recommended values threshold above.
3. As shown in Table 2, all of the results for composite reliability (CR), which measures the degree to which items are free from random error and therefore yield consistent results, are over 0.7, indicating that the scales have good reliability [53]. Specifically, all the standard loadings are over 0.7 and are significant at the 1% level.
4. In addition, as shown in Table 2, the average variance extracted (AVE) for each construct ranges from 0.59 to 0.87, which is over 0.5 and indicates that the scales have good convergent validities [54].

The composite reliability (CR) will be used to test the scales' reliability [53] and the average variance extracted (AVE) to test the convergent validates [54]. By comparing the square root of the AVE of each construct and its correlation coefficients with other constructs, the discriminant validity is examined and is shown in Table 3; all square roots of AVEs are bigger than the correlation coefficients of other constructs, indicating good discriminant validity.

## 3. Results

In total, three competing models are constructed to determine the best-fitting model for understanding the psychological mechanism of exercise behavior, namely, competing model 1(enjoyment + TPB model), competing model 2 (concentration + TPB model), and competing model 3 (enjoyment + concentration + TPB model). In competing model 1, enjoyment is added to TPB constructs by itself to explore the relationship between the two, In competing model 2, concentration is added to TPB constructs by itself to explore the relationship between them, In competing model 3, enjoyment and concentration are added into the TPB model at the same time to discuss the relationship between them. The path coefficients of the three competing models are shown in Table 4.

### 3.1. Competing Model 1

For competing model 1, Figure 2 shows the estimated model (enjoyment-TPB model) with standardized path coefficients. The fit measures indicate that the proposed model fits the data well: *χ*2/df = 1.829, RMSEA = 0.058, GFI = 0.927, CFI = 0.973, and NFI. = 0.943, IFI = 0.974.

Regarding the psychological flow variables, the hypothesized paths from enjoyment to attitude, norm, PBC, and exercise behavior except intention were significant. The enjoyment was significant and positively related to attitude (*β* = 0.443, *P* < 0.01), norm (*β* = 0.261, *P* < 0.001), PBC (*β* = 0.435, *P* < 0.01), and behavior (*β* = 0.149, *P* < 0.01). The enjoyment was the strongest predictor of attitude(*r*^2^ = 0.20), followed by PBC(*r*^2^ = 0.19), and NORM (*r*^2^ = 0.07) was the weakest. In addition, the enjoyment also has a significant indirect effect on exercise behavior via the attitude, norm, and PBC separately and then via intention. The direct relationship between enjoyment and intention is not significant(*β* = 0.04). These constructs jointly explained 25.3% of the variance in exercise behavior (*R*^2^ = 0.25.3) and 70.1% of the variance in intention (*R*^2^ = 0.70.1).

### 3.2. Competing Model 2

For competing model 2, Figure 3 shows the estimated model (concentration-TPB model) with standardized path coefficients. The fit measures indicate that the proposed model fits the data well: *χ*2/df = 2.109, RMSEA = 0.067, GFI = 0.918, CFI = 0.968, NFI. = 0.941, and IFI = 0.968.

The hypothesized paths from concentration to attitude, norm, and PBC except intention and exercise behavior were significant. The concentration was significant and positively related to attitude (*β* = 0.222, *P* < 0.01), norm (*β* = 0.170, *P* < 0.001), and PBC (*β* = 0.273, *P* < 0.01). The concentration was the strongest predictor of PBC (*r*^2^ = 0.07), followed by attitude (*r*^2^ = 0.05), and norm (*r*^2^ = 0.03) was the weakest. In addition, the concentration also has a significant indirect effect on exercise behavior via the attitude, norm, and PBC separately and then via intention. However, the direct relationship between concentration and intention (*β* = 0.06) and between exercise behavior (*β* = 0.01) is not significant in this research. These constructs jointly explained 23.9% of the variance in exercise behavior (*R*^2^ = 0.23.9) and 70.2% of the variance in intention (*R*^2^ = 0.702).

### 3.3. Competing Model 3

For competing model 3, it is to include enjoyment and concentration into the TPB model at same time to discuss the relationship between them.  Figure 4 shows the estimated model with standardized path coefficients. The fit measures indicate that the proposed model fits the data well: *χ*2/df = 1.754, RMSEA = 0.055, GFI = 0.909, CFI = 0.966, and NFI. = 0.926. These constructs jointly explained 25.2% of the variance in exercise behavior (*R*^2^ = 0.25.2) and 70.2% of the variance in intention (*R*^2^ = 0.70.2).

The hypothesized paths from enjoyment to attitude, norm, PBC, and exercise behavior except intention were significant. The enjoyment was significant and positively related to attitude (*β* = 0.434, *P* < 0.01), norm (*β* = 0.232, *P* < 0.001), PBC (*β* = 0.395, *P* < 0.01), and exercise behavior (*β* = 0.14.5, *P* < 0.01). In addition, the enjoyment also has a significant indirect effect on exercise behavior via the attitude, norm, and PBC separately and then via intention. However, the direct relationship between concentration and intention and with behavior is not significant. In addition, all the hypothesized links of concentration between TPB variables and between exercise behavior were not supported in competing model 3.

The three competing structural models all include TPB models. As expected, intention is found to have a significant predicting effect on actual exercise behavior (*β* = 0.43, 0.49, 0.43) in three competing models, revealing the strong predictive power of intentions with regard to actual exercise behavior. All the three TPB antecedents, the attitude (*β* = 0.223, 0.218, 0.220), norm (*β* = 0.239, 0.238, 0.238), and PBC(*β* = 0.470, 0.475, 0.473), have a significant positive effect on intention. In addition, the attitude, norm, and PBC also have significant indirect effect on exercise behavior via intention. PBC is the most powerful predictor of intention(*β* = 0.470, 0.475, 0.473), and the direct relationship between PBC and exercise behavior is not significant(*β* = 0.12, 0.123, 0.127). These constructs jointly explained 23.8–25.3% of the variance in exercise behavior (*R*^2^ = 0.253, 0.238, 0.252) and 70.2% of the variance in intention (*R*^2^ = 0.702, 0.703, 0.708).

### 3.4. Comparison of the Competing Models

After the model evaluation results were finished and satisfied, this research conducted a two-step comparison of a nested model and a non-nested model to determine the better model among the three models.

#### 3.4.1. First Step: Nested Model Comparison between Competing Model 1 and Competing Model 3

In this study, since competing model 1 and competing model 3 are classified as nested structures, we using the chi-square difference test to compare competing model 1 and competing model 3 to determine which model performs more effectively and better. In Table 4, the goodness-of-fit indices indicate no significant difference between competing model 1 and competing model 3. Moreover, the chi-square difference between the two models was -93.894 (∆*χ*2 = 149.886–243.780), much lower than the critical value of 7.815 for three degrees of freedom, showing that the competing model 1 (restricted model) is not significantly different from the competing model 3 (freely estimated model). That is to say, when the three nonsignificant direct hypothetical paths are excluded (concentration ⟶ attitude, concentration ⟶ SN, and concentration ⟶ PBC), the structure of competing model 1 is identical to that of competing model 3, and the explanatory power of competing model 3 (*R*^2^ = 0.252) is slightly lower than that of competing model 1 (*R*^2^ = 0.253). Therefore, competing model 1 is considered the better-fitting model than competing model 3.

#### 3.4.2. Second Step: Non-Nested Model Comparison among Competing Model 1 and Competing Model 2

This study conducted a non-nested model comparison among competing model 1 and competing model 2 according to the results of the first step. For this type of model comparison, the most common statistical test is *χ*2/d.f. analysis. As shown in Table 4, various fit measures indicate that all two models have a good fit to the data, and overall, competing model 1 has a better fit than those of both competing model 2. For competing model 1, the AIC was 227.886, the BIC was 364.910, and the ECVI was 0.923. For competing model 2, the AIC was 248.852, the BIC was 385.876, and the ECVI was 1.007. Because lower values of these criteria indicate a better fit of the model, these results indicate a preference for competing model 1 over competing model 2. Finally, the results indicate that all two models provide high explanatory power for exercise behavior. Competing model 1 provides somewhat greater explanatory power (*R*2 = 0.253) relative to competing model 2 (*R*^2^ = 0.252). So, competing model 1 is superior to competing model 2.

In short, the results suggest that of the three models, competing model 1 is superior to competing model 2 and competing model 3, meaning that competing model 1 is the best-fitting model for explaining the exercise behavior.

## 4. Discussion

### 4.1. TPB

For TPB parts in three competing models, as expected, intention is found to have a significantly positive effect on actual exercise behavior, revealing the strong predictive power of intentions with regard to actual exercise behavior. It is worth noting that the intention was the strongest and significant direct predictor of exercise behavior, meaning university students who have the motivation to exercise are more likely to show the exercise behavior. Consistent with previous studies [55], this result confirmed that intention to exercise is the overall motivation for universities to involve in exercise. Additionally, three competing models explained 70–71% of the variance in intention to exercise, while PBC, attitude, and norm were the powerful predictors. This variance is basically in accordance with between 28% and 68% of the variance in intention showed in related previous research studies (e.g., [25,55–57].

All the three TPB antecedents, the attitude, norm, and PBC have a significant positive effect on intention; in addition, the attitude, norm, and PBC also have a significant indirect effect on exercise behavior via intention, which indicates that the greater a university student's attitude and PBC is toward exercise, the greater the likelihood that they intend to show the exercise behavior. In the same way, the more subjective norms university students feel, the more likely they are intended to participate in exercise behavior, which is consistent with the previous research [1,11,38].

According to Ajzen [28], the strength or weakness in the relationship of PBC and intention relationship is dependent on the situation nature and behavior type. PBC is the most powerful predictor of intention, and the direct relationship between PBC and exercise behavior is not significant, which is not consistent with the previous research [1]. When perceived behavioral control accurately reflects the degree of actual environmental obstacles or resistance to participating behaviors, it can be used as a “proxy” measure of actual control and directly affect behaviors without the intermediary role of behavioral intention [37]. At present, Chinese universities provide very good material and institutional conditions for the exercise behavior of university students, and there is basically no obstacle from the actual environment. Therefore, the direct effect of PBC on exercise behavior is not significant, which is consistent with the previous research results of Chinese scholars [38,58]. In addition, this result confirmed the findings that the people's perceptions of control over dispositional resources do to some extent reflect their ability to abstain from behavior [55].

Consistent with the previous research studies [59], the subjective norm also predicted intention to exerciser. Therefore, a significant relation between norm and intention indicates promote and encourage for exercise behaviors. Thus, the results demonstrate that students are under influence of motivations, they may have the urge to exercise, and the opinions of important people to them might encourage their exercise behavior. Moreover, it means university students may join the exercise behavior when they perceive to receive social positivity and encouragement for exercise behavior and important others would exercise themselves.

### 4.2. Competing Model 1

For competing model 1, enjoyment has significant predictive effects on the three antecedents of TPB, respectively, and the exercise behavior is predicted through the continuous mediating effects of TPB's three antecedents and intention by enjoyment. In addition, enjoyment also has the direct predictive effect on exercise behavior, which is consistent with previous studies [19,30].

The research result of the relationship between enjoyment and TPB variables shows that enjoyment can significantly, directly, and independently predicting attitude, norm, and PBC towards exercise behavior. Among the three antecedent variables of TPB, enjoyment has the strongest predictive power on attitude, followed by PBC, and the least on NORM, which is consistent with the previous research conclusion [30].

The direct predictive effect of enjoyment on exercise behavior, which is consistent with previous studies [30, 60]. Gardner and his colleagues [38] also support the use of enjoyment and intention as predictors of sports participation behavior. These findings suggest that sensation may play a more pervasive role in motor behavior than thought. The direct influence of enjoyment on sports behavior means that when enjoyment is stimulated by motivation, university students' sports behavior may acquire the power of intention. These results indicate that the intervention of exercise behavior of university students can be considered through flow, especially the link of enjoyment, and the specific details need to be further studied.

The predictive power of enjoyment to attitude is the biggest, which is consistent with the previous research conclusion. Ginis et al. [39] found enjoyment-mediated changes in attitudes toward physical activity. His finding bolsters notion that affective reactions to an object or an action can shape attitudes toward it [40]. This is an important finding, given that direct experience is considered the strongest determinant of attitude within the theory of planned behavior. Exercise enjoyment has been theoretical [61]. The observed mediational relationship between exercise, enjoyment, and attitudes suggests that there is utility in further study of enjoyment within a theory of planned behavior framework.

The predictive power of enjoyment to PBC is basically equal to that of enjoyment to attitude, which is consistent with the previous research conclusion. Dishman and his colleagues believed that an additional, indirect effect of physical activity enjoyment on physical activity operated by an influence on self-efficacy. This explanation is consistent with Dishman and his colleagues' [41] finding that enjoyment's effects on physical activity are mediated partially by changes in self-efficacy, a control construct that is conceptually similar to PBC [43]. Therefore, in an enjoyment disposition, if an exerciser has a strong intention to perform an exercise behavior, he may feel to have the necessary resources and skills to perform the behavior [44]. In other words, enjoyment increases a person behavioral control and has been found to positively influence perceived behavior control [32].

Research studies investigating how enjoyment is related to intention and behavior through subjective norm are rare. Even so, Charles Atombo and his colleagues (2017) believed that the tendency of drivers in the enjoyment state to speed is influenced by the subjective norms of important individuals (e.g., family, friends, spouse, police) and that is subjective norms [45]. Similarly, in physical exercise, the enjoyment of this positive emotional experience can be influenced by the opinions of the important people around you. The results of this study also support the view above that enjoyment also has a significant predictive effect on subjective norms.

### 4.3. Competing Mode 2

For competing model 2, concentration has significant predictive effects on the three antecedents of TPB, and the exercise behavior is predicted through the continuous mediating effects of TPB's three antecedents and intention by concentration. In addition, concentration also has no direct predictive effect on intention and exercise behavior, which is consistent with previous studies [30].

The research result of the relationship between concentration and TPB variables shows that concentration was significantly and directly, but independently associated with the attitude, norm, and PBC towards exercise behavior. Among the three antecedent variables of TPB, concentration has the strongest predictive power on PBC, followed by Attitude, and the least on NORM, which is consistent with the previous research conclusions [30].

Similar with enjoyment, both as a factors of flow, the concentration has been believed to be positively correlated with attitude and intention [31]. It may be based on the facts that individuals are more likely to be motivated to continue or repeat any activity that is enjoyable as compared to the same activity, which is not enjoyable. Moreover, in the pursuit of a goal, a person must concentrate on the task and forget everything [46]. All these studies have evidenced that flow constructs are capable of predicting intention and behavior. A current study also examined the causal relationship between flow constructs and PBC [32] and found concentration to be positively related to PBC constructs (self-efficacy and controllability). A person's concentration could also affect exercise intentions and behavior when perceived other important people are against or in support of exercise [44]. This is consistent with the conclusion of this study that there is a chain mediating effect between concentration, subjective norms, exercise intention, and exercise behavior.

### 4.4. Competing Model 3

For competing model 3, when enjoyment and concentration are considered simultaneously in the TPB model, contrary to a previous study [31] and expectation, although enjoyment still shows the significant direct predicting effect on TPB antecedents and exercise behavior and shows a significant indirect predicting effect on behavior by the continuous mediation of TPB antecedents and intention, the relationship between concentration and three TPB antecedents of TPB and intention in competing model 3 was found not significant, which are partly the same with another previous research [30]. Therefore, it can be concluded that enjoyment and concentration as factors of flow all can independently and significantly predict the TPB structure by itself. However, the enjoyment explains basically the same position of the variance of TPB constructs with concentration do and enjoyment explained enough variance more than concentration do in competing model 3. In addition, there is a high correlation between them both as factors of the flow. Therefore, when the two are estimated in the same model, concentration is not significant relative to enjoyment. These findings indicate that enjoyment is more important than concentration and better than concentration in predicting TPB, and concentration is not a direct determinant of intention and is likely not direct related to exercise behavior, at least in the exercise behavior research context. When it comes to the intervention of exercise behavior of university students, enjoyment factor should be taken into more consideration than concentration.

### 4.5. Competing Model Discussion

Based on the conclusion of three competing models, enjoyment and concentration all significantly and directly, but independently predicted the attitude, norm, and PBC, and predicted the exercise behavior via the mediation of TPB. This suggests that the flow structure may be an important predictor of university students' exercise behavior in exercise environments.

Through the comparison of three competing models, competing model 1 (enjoyment + TPB model) is superior to competing model 2 (concentration + TPB model) and competing model 3 (enjoyment + concentration + TPB model), meaning that the enjoyment + TPB model is the best-fitting model for explaining the exercise behavior. The enjoyment + TPB model explains the variance of exercise behavior best and has the highest degree of fitting with data, which can explain the interaction mechanism of flow and TPB to the maximum extent in the most concise form. This confirms the importance of enjoyment factor in flow constructs and in the field of exercise behavior research.

So, through the comparison of three competing models, enjoyment was again shown to be important in the exercise behavior research context. Exercisers with higher levels of enjoyment-seeking are more likely to show better behavior. According to a previous study of [55], this result may mean that university students may intend to exercise because they feel exercise will be enjoyable, even though they know exercise may be tiring. Exercisers who are under the influence of enjoyment to enjoy the experience of exercise behavior may have more illustrative encouragement with regard to exercise. Therefore, in addressing measures to promoting exercise behavior, it is important not to focus only on what the exerciser intends to do, but also on the exerciser's emotions as possible factors that can influence behavior.

When it comes to the intervention of exercise behavior of university students, enjoyment factor should be taken into more consideration. Thus, the conclusion drawn from this study is that the containing of flow constructs, especially enjoyment, helps increase the explanation exercise behavior when designing measures (e.g., education and training) for promoting or changing behaviors.

### 4.6. General Discussion

The purpose of this study is to extend the planned behavior theory (TPB) to explain the intention and behavior of Chinese university students by adding the variables of flow and to evaluate the factors that are important to explain intention and behavior.

The flow explored in this study consisted of enjoyment and concentration, and the TPB consisted of attitude, subjective norm, perceived behavior control, and exercise intention. The study result shows that all the hypothesized links of enjoyment between TPB factors and between exercise behavior were supported in competing model 1. However, there are some differences about concentration. All the hypothesized links of concentration between TPB factors were supported, except for the links between concentration and exercise behavior in competing model 2. But all the hypothesized links of concentration between TPB variables and between exercise behavior were not supported in competing model 3.

Generally, the current results provide important support for the predicting power of the combined TPB and flow variables. Three competing models all can significantly predict behavior and accounted for more than 24% of the variance in exercise behavior, and intention, concentration, and enjoyment all can significantly predict exercise behavior. These results are basically consistent with the previous research results that add variables into TPB to predict exercise behavior [25, 55–57]. Thus, the conclusion drawn from the present study is that the inclusion of flow constructs, especially enjoyment, helps deepen the explanation of exercise behavior.

In total, the variance explained in the intention and behavior by the integrated model in this research showed the importance of integrated model constructs in understanding exercise intention and behavior. The findings suggest the need for appropriate interventions, aimed at beliefs influencing the exercise behaviors of exerciser. Furthermore, enjoyment is of considerable importance to the participant's exercise behavior. In China, a lots of the university students, especially women, do not like exercise or have bad exercise behavior. The present findings imply that there is strong justification for developing university interventions that deal with the variables of flow and TPB factors toward exercise, aimed at university students. This is because flow and TPB factors were significant predictors of exercise behavior and had a significant total effect on exercise behavior. These research studies therefore provide insights to better understand the exercise behavior of Chinese university students as well as useful information for designing exercise interventions and developing university students' education and training. However, how to make the best use of the emotional factors or intrinsic motivation relating university students' sports behavior and apply them to practice is a new problem and challenge, which also provides research direction for future.

### 4.7. Limitation and Suggestion for Future Study

#### 4.7.1. Limitation

Firstly, this study is conducted on Chinese university students. As only Chinese university students are used as research objects, the survey data have certain limitations. Therefore, direct application of the results to other countries or populations may be biased, because “every country and population has its own cultural issues.” Different cultures evaluate and express psychological and behavioral factors differently. Secondly, flow is a multifaceted concept and that includes several dimensions. In this research, we only used enjoyment and concentration to measure the flow. In the future, flow-up studies can give more attention to this theory.

#### 4.7.2. Suggestion for Future Study

So far, the “gap” between intention and exercise behavior still exists in the studies on TPB and exercise behavior. It is suggested to continue to explore new variables to improve the predictive power of TPB.

In future studies, the moderating effects of exercise habit, exercise level, personality, and other factors on this research model can be explored through multigroup comparative analysis, so as to gain a deeper understanding of exercise behavior and its psychological mechanism [62, 63].

## Figures and Tables

**Figure 1:** Hypothesis model of the flow integrating theory of planned behavior.

**Figure 2:** Competing model 1: enjoyment + TPB mode.

**Figure 3:** Competing model 2: concentration + TPB model.

**Figure 4:** Competing model 3: enjoyment + concentration + TPB model.

**Table 1:** Descriptive statistical analysis of research objects.

		*N*	%
Gender	Male	165	66.5
	Female	83	33.5
Census register	City	112	45.2
	Country	136	54.8
Grade	Grade 1	55	22.2
	Grade 2	92	37.1
	Grade 3	64	25.8
	Grade 4	37	14.9
Total	248		100

**Table 2:** Confirmatory factor analysis.

Construct	Items	Loading	AVE	CR
Enjoyment	Enjoyment1	0.794	0.6183	0.8661
	Enjoyment2	0.756		
	Enjoyment3	0.831		
	Enjoyment4	0.762		

Concentration	Concentration1	0.731	0.6355	0.8739
	Concentration2	0.745		
	Concentration3	0.815		
	Concentration4	0.888		

Intention	Intention1	0.914	0.8672	0.9514
	Intention2	0.918		
	Intention3	0.961		

Attitude	Attitude1	0.806	0.5881	0.8105

	Attitude2	0.755		
	Attitude3	0.738		
PBC	PBC1	0.894	0.7608	0.9048
	PBC2	0.920		
	PBC3	0.798		

**Table 3:** Discriminant validity.

	1	2	3	4	5
Enjoyment	**0.786**				
Concentration	0.485	**0.797**			
Intention	0.391	0.266	**0.931**		
Attitude	0.439	0.225	0.735	**0.907**	
PBC	0.430	0.268	0.801	0.801	**0.872**

*Note.* Values in the diagonal (bolded) represent the square root of the AVE, whereas the off-diagonals are correlations between constructs.

**Table 4:** The estimated results of three competing models.

Path	Competing model 1: enjoyment + TPB model	Competing model 2: concentration + TPB model	Competing model 3: enjoyment + concentration + TPB model
Enjoyment-attitude	0.443^∗^		0.435^∗^
Enjoyment-norm	0.261^∗^		0.232^∗^
Enjoyment-PBC	0.435^∗^		0.395^∗^
Concentration-attitude		0.222^∗^	0.014
Concentration-norm		0.170^∗^	0.058
Concentration-PBC		0.273^∗^	0.083
Attitude-intention	0.223^∗^	0.218^∗^	0.220^∗^
Norm-intention	0.239^∗^	0.238^∗^	0.238^∗^
PBC-intention	0.470^∗^	0.475^∗^	0.473^∗^
Intention-behavior	0.429^∗^	0.488	0.431^∗^
Enjoyment-behavior	0.149^∗^		0.145^∗^
Goodness of fit index	CMIN/DF = 1.829 (*P* = 0.000); GFI = 0.927; IFI = 0.974; NFI = 0.943; CFI = 0.973; RMSEA = 0.058	CMIN/DF = 2.109 (*P* = 0.000); GFI = 0.918; IFI = 0.968; NFI = 0.941; CFI = 0.968; RMSEA = 0.067	CMIN/DF = 1.754 (*P* = 0.000); GFI = 0.909；IFI = 0.967; NFI = 0.926；CFI = 0.966; RMSEA = 0.055
Goodness-of-fit index for model comparison	ACMIN = 149.886 AIC = 227.886 BIC = 364.910 ECVI = 0.923	CMIN = 170.852 AIC = 248.852 BIC = 385.876 ECVI = 1.007	CMIN = 243.780 AIC = 345.780 BIC = 524.965 ECVI = 1.400
Explanatory power	0.253	0.238	0.252

## Data Availability

All the data contained in this study can be obtained by contacting the corresponding author. Readers can also inquire part of the original data and the results of data processing in this paper.
